# Profiling of T cell repertoire in peripheral blood of patients from type 2 diabetes with complication

**DOI:** 10.1186/s12865-024-00601-7

**Published:** 2024-01-31

**Authors:** YongHui Yin, YingLi Sheng, Shuo Gao, JinTao Zhang, WenKuan Wang, YingJun Liu, TingTing Xu, Yi Zhang

**Affiliations:** 1 Shandong University of Traditional Chinese Medicine Affiliated Hospital, Jinan, Shandong 250014 China; 2 Shandong University of Traditional Chinese Medicine, 203, Administrative Building, 4655 University Road, Changqing District, Jinan, Shandong 250035 China

**Keywords:** Type 2 diabetes, Large cardiovascular complications, Kidney complications, T-cell receptor repertoire, High-throughput sequencing

## Abstract

**Purpose:**

More than 90% of patients with diabetes worldwide are type 2 diabetes (T2D), which is caused by insulin resistance or impaired producing insulin by pancreatic β cells. T2D and its complications, mainly large cardiovascular (LCV) and kidney (Ne) complications, are the major cause of death in diabetes patients. Recently, the dysregulation of peripheral T cell immune homeostasis was found in most T2D patients. However, the characteristics of T-cell receptors (TCR) remain largely unexplored in T2D patients.

**Patients and methods:**

Here we investigated the TCR repertoire using high-throughput sequencing in peripheral blood collected from T2D patient with (8 LCV and 7 Ne) or without complications.

**Results:**

Our analysis of TCR repertoires in peripheral blood samples showed that TCR profiles in T2D patients with complications tended to be single and specific compared to controls, according to the characteristics of TCR repertoire in V-J combination number, diversity, principal component analysis (PCA) and differential genes. And we identified some differentially expressed V-J gene segments and amino acid clonotypes, which had the potential to contribute to distinguishing T2D patient with or without complications. As the progression of the disease, we found that the profiling of TCR repertoire was also differential between T2D patients with LVD and Ne complications base on this pilot analysis.

**Conclusion:**

This study demonstrated the protentional unique property of TCR repertoire in peripheral blood of T2D patient with and without complications, or T2D patients with LVD and Ne complications, which provided the possibility for future improvements in immune-related diagnosis and therapy for T2D complications.

## Introduction

Diabetes mellitus (DM) is a global health problem, which affect approximately 8.3% of adults worldwide, expected to reach 10.1% of adult population in 2035 [1]. There are two major types of diabetes, type 1 diabetes (T1D) and type 2 diabetes (T2D). More than 90% of patients with diabetes worldwide are T2D, which is caused by insulin resistance or impaired producing insulin by pancreatic β cells [2]. The chronic insulin resistance in T2D patients for a long term could result in the development of several complications, including macrovascular disorder such as atherosclerosis, as well as microvascular disorder such as nephropathy, neuropathy, and retinopathy [3]. DM and its complications accounts for 5.2% of all deaths, and is the fifth principal death cause worldwide. In T2D patients, morbidity and mortality from cardiovascular complications are the highest, and kidney complications are highly prevalent in Asia patients [4]. Hyperglycemia in diabetes is thought to cause dysfunction of the immune response, which fails to control the spread of invading pathogens in diabetic patients.

Recently, studies had suggested that adaptive immune system, especially T cells, played a vital role in the development of T2D. Studies have shown that diabetic patients, the levels of naive T-cells and TCRVβ repertoire diversity were reduced, but the number of effector T cells was elevated [5]. Due to the variety of foreign antigens, the quantity and diversity of TCR repertoire determines the T cell-mediated immune response to a given antigen [6]. The diversity of TCR repertoire is mainly determined by complementary determination region 3 (CDR3) generated by genomic rearrangement of the variable (V), diversity (D), and joining (J) regions [7]. Therefore, highthroughput sequencing (HTS) of CDR3 region on the TCR could facilitate our understanding of the adaptive immune state of the organism. Recently, several studies have illuminated that CDR3 diversity of TCR can serve as a relatively stable biomarker, contributing to early disease diagnosis, efficacy monitoring, and prognostic evaluation [8, 9]. However, few studies compared the differences of TCR repertoire in T2D patients with or without complications.

In the present study, we analyzed the difference in composition of TCR repertoire in peripheral blood of T2D patients with or without complications. We hope that TCR repertoire analyzing will be helpful to determining the immune status and contribute to differential diagnosis, efficacy assessment, and prognosis prediction.

## Material and methods

### Patient enrollment

Large cardiovascular complications (LCV), and kidney complications (Ne).Screening 30patients as the research objects, according to the presence or absence of complications were divided into two groups from Shandong University of Traditional Chinese Medicine Affiliated Hospital.Clinical data was extracted from our medical records, including gender, age, BMI, fasting blood glucose (FBG), glycosylated hemoglobin (HbA1c), total cholesterol (TC), triglyceride (TG), high density lipoprotein-cholesterol (HDL-C), low-grade lipoprotein cholesterol (LDL-C), comorbidity information, complications information, current therapy and family history of diabetes. The Shandong University of Traditional Chinese Medicine Affiliated Hospital's Ethics Committee examined and approved each procedure. Every patient’s completed an informed consent form in accordance with the Institutional Review Board-approved procedure (registration number:(2018) No. 025 Ethics-KY).

### Sample processing and TCR sequencing

Venous blood samples were collected in EDTA vacutainer tubes at volumes greater than 2 mL. Total RNA was extracted from samples using RNA simple Total RNA Kit (DP419, Tiangen Biotech, Beijing, China).In this study, the minimum concentration of total RNA was 1008 ng, and all samples were qualified base on the threshold of RNA input (100 ng). The concentrations of total RNA were evaluated using a NanoDrop ND-2000 spectrophotometer (Thermo Scientific, UK). cDNA synthesis and multiplex PCR amplification of all possible rearranged TCR β-chain sequences were performed together using the Immune Repertoire Library Preparation Kit (Geneway, Jinan, China) following a protocol described in a previous study [10]. TCR libraries were sequenced on the DNBSEQ-T7 platform (MGI, Shenzhen, China), generating paired-end short reads with 150 bp in length.

### Sequencing data preprocessing

The sequencing data were stored in FASTQ format, in which raw reads were demultiplexed according to the sequences of index primers corresponding to different samples. The low-quality sequences were discarded for quality control and the remainders were mapped into V, D, and J gene segments of TCR β-chain using the MiXCR software (version 3.0.6) with default parameters for both sequencing alignment and clonotype assembly [11]. TCR reference gene data were downloaded from the IMGT database (http://www.imgt.org/vquest/refseqh.html). The frequency of each TCRβ clonotype was further converted into rpm (reads per million) for standardization.

### Availability of data and materials

The raw datasets generated and analyzed during the current study are available in the NCBI-SRA repository, which can be accessed at the Sequence Read Archive of National Center for Biotechnology Information (NCBI, PRJNA980965).

### Statistical analyses

The data were analyzed with R software (version 4.0.2). Continuous data were presented as means ± standard deviation while categorical variables were presented as number and percentage. For continuous variables, Student's t-test or Wilcoxon rank-sum test was used for comparison between the two groups. For categorical variables, Fisher's exact test was performed. *P* < 0.05 was considered as the threshold of statistical significance. The diversity of samples were evaluated base on D50 Diversity index and Gini index. The diversity from the cumulative 50% of the total CDR3 detected in the sample was measured using the D50 index [12]. The Gini index ranged from 0 to 1,and was calculated by “ineq” package in R [13].

## Results

### Characteristics of participants

During the research period, 30 T2D patients and their blood samples were enrolled. These samples were qualified and underwent TCR sequencing, and grouped base on their clinical backgrounds. Finally, we investigated the TCR repertoire using high-throughput sequencing in peripheral blood collected from 30 T2D patient with (8 LCV and 7 Ne) or without (15 None) complications. The detail infomations of each sample was shown in Table 1.

**Table 1:** Clinical Information for Samples

SampleID	Gender	Age	BMI	Comorbidity information	Complications information	Current therapy	Family history of diabetes	fasting blood glucose (FBG)	glycosylated hemoglobin (HbA1c)	total cholesterol (TC)	triglyceride (TG)	high density lipoprotein-cholesterol (HDL-C)	low-grade lipoprotein cholesterol (LDL-C)
S3_12	female	59	26.56	YES	LCV	NA	YES	4.73	5.6	4.31	1.32	1.04	2.63
S3_14	male	76	23.85	YES	LCV	Isophane Protamine Biosynthetic Human Insulin Injection, Metformin, Acarbose Tablets	NO	18.84	10.8	5.73	1.56	1.13	3.91
S3_17	male	63	25.2	TES	LCV	Metformin 0.5g bid;Dapagliflozin 10mg qd	YES	6.6	6.3	6.24	0.95	1.59	4.19
S3_18	female	63	25	YES	LCV	Protamine Zinc Insulin Injection, acm: 16u, acv: 14u	YES	5.59	6.9	6.29	0.43	1.29	1.56
S3_21	male	59	22	YES	LCV	Metformin 0.5g bid;Acarbose Tablets 50mg tid;Insulin Aspart 30 Injection	NO	7.84	7.2	3.75	1.03	1.02	2.37
S3_22	male	47	26.8	YES	LCV	Metformin 0.5g bid;Dapagliflozin 10 mg qd	YES	6.49	5.7	4.2	0.56	1.36	2.47
S3_23	male	54	23	YES	LCV	Metformin 0.5 g bid;Acarbose Tablets 50 mg tid	YES	7	7.5	5.9	3.65	0.76	3.75
S3_2	male	59	26.2	YES	LCV	Metformin 0.5g bid;Empagliflozin 10mg qd	YES	5.69	6.1	4.78	0.61	1.58	2.64
S2_14	male	42	22	YES	NE	Metformin 0.5g bid;Dapagliflozin 10mg qd;Acarbose Tablets acv 50mg	YES	9.93	9.2	5.25	0.66	1.44	3.55
S3_19	male	68	24	YES	NE	Metformin 0.5g bid;Dapagliflozin 10mg qd;Glimepiride 10mg qd	YES	8.3	7	4.12	2.32	1.2	3.67
S3_20	male	61	21	YES	NE	Metformin 0.5g bid;Dapagliflozin 10mg qd	YES	8.56	7.5	3.19	1.12	0.72	1.95
S3_24	female	70	24	YES	NE	Metformin 0.5 g bid;Dapagliflozin 10 mg qd	NO	6.91	7.1	5.7	1.17	1.51	3.38
S3_5	female	73	24.6	YES	NE	Metformin 0.5g bid;Dapagliflozin 10mg qd;Insulin Glargine Injection qn 16u	YES	9.25	6.6	3.44	0.8	1.65	1.47
S3_6	male	66	21	YES	NE	Dapagliflozin 10mg qd;Acarbose Tablets 50mg tid	YES	8.46	7.4	3.33	0.94	1.22	1.78
S3_8	female	65	20.6	YES	NE	Insulin Aspart 30 Injection acm 22u;acv 20u	YES	8	6.7	4.52	2.45	1.35	2.78
GuoLei	male	40	27.08	NO	NO	NA	NO	16.02	10.4	9.65	5.55	6.36	1.12
S2_10	female	54	20.6	NO	NO	NA	YES	8.9	7.1	4.56	0.69	1.63	2.68
S2_11	female	38	23.15	NO	NO	Metformin 0.5g bid;Acarbose Tablets 50mg tid	YES	8.67	8.9	4.39	0.88	2.9	1.25
S2_15	male	29	24.5	NO	NO	Insulin degludec 14u;Insulin Aspart Injection acm、acl、acv 6u	NO	12	5.4	3.4	0.52	1.59	1.28
S2_17	female	39	20.6	NO	NO	Metformin 0.5g bid;Dapagliflozin 10mg qd	YES	6	6.4	6.57	1.8	0.99	4.61
S2_18	male	30	26.7	NO	NO	Metformin 0.5g bid;Polyethylene Glycol Loxenatide Injection 0.1g qw	YES	11.1	8.1	4.84	4.28	0.99	2.17
S2_19	male	21	24.7	NO	NO	NA	NO	5.35	8.5	4.11	1.2	0.78	2.67
S2_3	male	35	40.54	NO	NO	Linagliptin 5mg qd;Liraglutide Injection 0.6mg qd	YES	12.34	10.8	3.5	6.18	0.99	4.01
S2_4	male	41	22.4	NO	NO	Metformin 0.5g bid;Dapagliflozin 10mg qd	YES	9.57	7.3	4.77	0.73	1.54	3.1
S2_6	female	51	23.65	NO	NO	Metformin 0.5g bid;Empagliflozin 10mg qd;Glimepiride 1mg qd	YES	16.07	8.5	5.21	2.78	1.24	3.09
S2_8	male	42	22.43	NO	NO	NA	NO	7.75	7.9	5.33	2.46	1.02	3.3
S2_9	female	36	24.15	NO	NO	Metformin 0.5g bid;Dapagliflozin 10mg qd	YES	9.23	8.4	5.38	1.44	1.33	3.89
S35_1	male	62	24.8	NO	NO	Metformin 0.5g bid;Dapagliflozin 11mg qd	NO	6.96	6.06	1.79	1.08	3.99	1.28
S134	female	38	23.45	NO	NO	Metformin 0.5g bid;Dapagliflozin 12mg qd	YES	7.37	8.4	5.78	1.69	0.89	4.01
S180	female	69	24.46	NO	NO	NA	YES	7.83	7.8	4.12	1.43	0.95	2.54

### The basic characteristic of TCR repertoires in T2D patients with or without complications

We performed TCR repertoire sequencing analysis of peripheral blood in T2D patients with or without complications (complications group and control group). We assembled the immune sequences and identified the V-J combinations at the transcription level. The results showed that the quantity of V-J combinations identified had a decreased trend in complications group than control group, but there was no statistical significance (Fig. 1A). We further performed Principal Component Analysis (PCA) on the V-J combination frequency profile. As shown in the PCA plot (Fig. 1B), a difference was found between complication group and control group. PCA of complication group was more loose than the control group, and showed a more broad spectrum of immune defense characteristics. TCR expression profiles were subsequently analyzed to assess their systemic immune responses.

**Fig. 1:** The quantity of CDR3 sequences number and diversity analyses between complication and none-complication in T2D. **A** Box plot of the quantity of CDR3 sequences numbers. **B** The PCA plot for TCR profiles. **C** Diversity analysis of D50 diversity index. **D** Diversity analysis of Gini index. Groups were compared using unpaired Student 's t-test. Red indicated the complication group, blue indicated the none-complication group

We calculated the D50 Diversity and Gini indexes to estimate the diversity of TCR clonotypes in each sample, which were not relevant to the variation of sample sequencing depth. The results showed that D50 Diversity index of complication group was lower than control group (Fig. 1C, *P* < 0.01). Moreover, Gini index showed that complication group was higher than control group (Fig. 1D, *P* < 0.01). The above data indicated that the diversity of TCR profiles decreased in complications group compared with control group.

### Different gene expression of V-J gene combinations in T2D patients with or without complications

We utilized the circos plots to show the average frequency usages of V/J gene combinations, which were found to be similar between complications group and control group (Fig. 2A,B). As figures showed, the V gene is more variable than the J gene in both groups and major genes clonotypes were same in both V and J genes.A total of 60 V and 14 J gene segments were identified in all samples. Compared with control group, complications group showed significantly higher percentage in the gene segments of TRBJ1-6 (Fig. 2C), and TRBV27, TRBV28, TRBV3-2 (Fig. 2D). The above data indicated that the differentially expressed V-J gene segments had the potential to be markers for T2D with or without complications.

**Fig. 2:** Character of V-J combinations between complication and none-complication in T2D. **A-B** V-J gene combinations circle plots of the complication group (**A**) and the none-complication group (**B**). The leftward side indicated J gene segments and rightward side indicated V gene segments. This plot showed the situation of V/J gene combinations. The length of sectors represents the relative usage frequency of the V genes or the J genes. The width of the links connecting the V genes and the J genes represents the relative usage frequency of the V/J combinations. **C-D** Bar plots showed differential gene segments of J gene segments (**C**) and V gene segments (**D**) between complication and none-complication groups’ individuals. The asterisks meant *P* < 0.05, red was the complication group and blue was the none-complication group

### Different amino acid clonotypes in T2D patients with or without complications

We further analyzed and compared the abundance of CDR3 sequences between complication group and control group. There was 50,863 up-regulated and 44,628 down-regulated CDR3 sequences (Fig. 3A,B). Also, we analyzed the differential expression of amino acid clonotypes. We found there were 25 differentially expressed amino acid clonotypes, in which 8 were up-regulated and 17 were down-regulated (Fig. 3C), which had the potential as the diagnostic marker of T2D patients with or without complications in the peripheral blood. Their sequences were presented in Fig. 3C.

**Fig. 3:** Character of differential CDR3 sequences. **A** The volcano map showed information on differentially expressed amino acid CDR3 sequences between complication and none-complication groups. The yellow dots were difference sequences with increasing abundances, while the blue dots were difference sequences with decreasing abundances. **B** Part of the differentially expressed amino acid CDR3 sequences of complication and none-complication groups were displayed in this scatter plot, the red dots were difference sequences. **C** Part of the differentially expressed amino acid CDR3 sequences of complication and none-complication groups were displayed in this heat map

### The characteristic of TCR repertoires in T2D patients with LVD or NE complications

Finally, we analyzed the characteristics of TCR repertoires in T2D patients with LVD or NE complications. The data showed that the quantity of V-J combinations in patients with LVD was more than ones with Ne, but there was no statistically significant (Fig. 4A). Then we performed PCA on the V-J combination frequency profile of patients with LVD or Ne, which was also able to distinguish between the two groups (Fig. 4B). The D50 Diversity and Gini indexes showed that the diversity of TCR composition in the group with LVD tended to increase over the group with Ne, but it was not statistically significant (Fig. 4C,D). To analyse the specificity of immune sequence abundance in patients with LVD or Ne, we found that high abundance sequence in patients with LVD appeared to be more than patients with Ne (the large color chip represented high abundance of this sequence) (Fig. 4E,F).

**Fig. 4:** Analysis of LVD and Ne groups. **A** Box plot of the quantity of CDR3 sequences numbers. **B** The PCA plot for TCR profiles. **C** Diversity analysis of D50 diversity index. **D** Diversity analysis of Gini index. Groups were compared using unpaired Student 's t-test. **E–F** treemap of module CDR3 sequences abundances in LVD group (**E**) and Ne group (**F**). **G-H** Logo plots showed consensus CDR3 motifs in LVD group (**G**) and Ne group (**B**), which illustrated amino acid CDR3 sequences whose expressed abundances were in top 50. Yellow indicated the LVD group, purple indicated the Ne group

We aligned the alignment of the top 50 abundant CDR3 sequences with the indicated length to make motif diagram. And the results showed that the motif in patients with LVD was different from patients with Ne (Fig. 4G,H), which suggested that selecting suitable amino acid sequence can effectively distinguish patients with LVD or Ne.

## Discussion

The pathogenesis of type 2 diabetes is insulin resistance and impaired islet β-cells function of the pancreas, accounting for approximately 90% of diabetic patients [14]. T2D patients have a greatly increased risk of cardiovascular, renal, brain complications and so on, among which cardiovascular complications caused the highest death in non-communicable diseases each year, with about 17.6 million people [15].

T1D is a typical organ-specific autoimmune disease in which the predominant immune response is mediated by T cells targeting the islet insulin-producing beta cells [16]. Previous investigators had analyzed the profiling of TCR repertoire in the peripheral blood of T1D patients by high-throughput sequencing, which could identify high abundance unique CDR3 amino acid sequence, providing support for specific TCR sequences as biomarkers and potential therapeutic targets [17].However, T2D is not an autoimmune disease, but recent researches showed that T cells could remove to the visceral adipose tissue (VAT) with a TCR repertoire changed, which demonstrated the expansion of antigen-special T cells were occurred in the VAT [18]. Another study showed that all Vβ families of resident T cells in the adipose tissue of T2D patients were significantly altered, suggesting that adipose tissue-resident T cells have specific restricted TCR repertoires [19]. TCR repertoire bias of tissue-resident T cells occurred frequently in organ-special autoimmune diseases [20], but was little reported in T2D patients.

An important feature of T2DM is chronic low-grade inflammation. Abnormal lipid metabolism can trigger chronic inflammatory response. This chronic inflammation may activate T cells, leading to abnormal immune responses.

In the present study, we analyzed the characteristics of the TCR repertoires in the peripheral blood of T2D patients with and without complications by using the techniques of high-throughput sequencing. We found that although there was no statistical difference in the quantity of V-J combinations between with and without complications, there was a decreasing trend in the patients with complications. PCA analysis had better distinguished the V-J combination frequency profile between T2D patients with and without complications. Both D50 Diversity and Gini indexes indicated that the diversity of TCR profiles decreased in complication group compared with control group. The above data indicate that the TCR repertoires of the complication group were significantly changed compared with the control group, which may be caused by the specific amplification of TCRs against antigen. Moreover, we screened out the specifically amplified fragments (TRBV27, TRBV28, TRBV3-2, and TRBJ1-6), and also 25 differentially expressed CDR3 sequences (8 up-regulated and 17 down-regulated) in the complication group, which had the potential to be a marker to predict complications of T2D patients.

To distinguish the profiles of TCR repertoires in T2D patients with different complications, we also analyzed and compared patients with LVD and Ne complications using high-throughput sequencing. We found that though there was no statistically significant, the quantity of V-J combinations in patients with LVD was more. And PCA on the V-J combination frequency profile could distinguish between LVD and Ne groups. Though there was no statistically significant, the diversity of TCR composition showed by D50 Diversity and Gini indexes in the group with LVD tended to increase. Moreover, the motif diagram of top 50 abundant CDR3 sequences showed that selecting suitable amino acid sequence can effectively distinguish patients with LVD or Ne complications.

TCR is a special marker that can determine the antigen specificity of specific T cells. Due to the development of sequencing methods and computational analysis techniques, TCR repertoires have become important drug candidates for a new generation of cell-free T lymphocyte markers. TCR biomarkers have the following advantages: 1) can be used for assays that do not require live T cells; 2) reduce intra- and inter-assay variability due to cell condition and operator performance; 3) newly developed high Throughput sequencing technology can detect rare and poorly responsive T cells.

Recently, high-throughput sequencing for TCR repertoires has been used to display T cells function in different conditions, such as immune diseases or cancers, suggesting that TCR repertoire may have the potential to reflect the immune status or serve as the prognostic marker [21]. Previous research on T-cell immunity and T1D evaluation was mainly carried out by methods such as Western blot, T cell proliferation, ELISPot and flow cytometry. These methods can distinguish T1D patients from normal controls, but their sensitivity and specificity are lower than using their own antibodies [22]. However, the immunoblot and T-cell proliferation assays usually required freshly isolated cells, which limited their application in the detection of a large number of clinical samples [23]. ELISpot and MHC polymer detection technologies could accurately identify target antigen epitopes and T lymphocyte phenotypes, but due to the limitations of sample conditions and HLA, multi-center studies were greatly hindered. However, through high-throughput sequencing for the profiling of TCR repertoires, researchers now can identify T cell clones, phenotypes, and the specific epitopes of T cells independent of HLA haplotypes [24].

There are still some limitations in this study that should be addressed. First, the current results are limited by the retrospective nature of our study. The relationship between TCR diversity and T2D development must be verified in prospective studies. Second, the relative small sample size might compromise the reliability of conclusions, which could be further confirmed by large-scale clinical cohorts. In addition, the causality and the predominant effects of TCR repertoire on T2D development remain unclear, and further study on the underlying immunological mechanisms is required.

There were several limitations of this study. First, all of the samples analyzed here were collected from one center, and the sample size was modest. Second, this analysis was based on bulk tissue samples, and these could not be used to identify immunological cells extracted from tissues. Finally, the specific function of each immune clonotype could not be identified. Therefore, large-scale investigations in the future are warranted.

In summary, this study revealed the divergence in TCR repertoire in T2D patients with (LVD or Ne) or without complications. Our findings provided novel insights into the role of T cell immunity in T2D incidence and progression, which may support the development of early diagnostic methods and targeting immunotherapies.

## Data Availability

All data generated or analyzed during this study are included in this published. article. The datasets used or analyzed during the current study are available. from the corresponding author on reasonable request.
